This article has been retracted.

# The Treatment Combining Antiangiogenesis with Chemoradiotherapy Impinges on the Peripheral Circulation Vascular Endothelial Cells and Therapeutic Effect in the Patients with Locally Advanced Nasopharyngeal Carcinoma

**DOI:** 10.1155/2022/1787854

**Published:** 2022-07-15

**Authors:** Xiuyun Gong, Limin Wang, Weili Wu, Yuanyuan Li, Jinhua Long, Xiaoxiao Chen, Xiuling Luo, Qianyong He, Ting Bi, Zhuoling Li, Yanan Luomeng, Feng Jin

**Affiliations:** ^1^Head and Neck Oncology, The Affiliated Cancer Hospital of Guizhou Medical University, The Affiliated Hospital of Guizhou Medical University, Guiyang 550004, China; ^2^Guiyang First People's Hospital, Guiyang 550002, China; ^3^Department of Oncology, Hainan Province Nongken General Hospital, Haikou 570100, China

## Abstract

This study was implemented for the evaluation on the circulating endothelial cells' (CECs) clinical significance in the locally advanced nasopharyngeal carcinoma treatment with endostatin-combined chemoradiotherapy. This study enrolled 47 patients with locally advanced nasopharyngeal carcinoma who were hospitalized from May 9, 2012 to March 10, 2013. These patients were split up into the observation group (25 patients) and control group (22 patients). Patients in the observation group received the endostatin combined with induction chemotherapy and subsequently with concurrent chemoradiotherapy with endostatin. Patients in the control group were treated with inductive chemotherapy followed by concurrent chemoradiotherapy. CECs in peripheral blood were conducted separately before or after inductive chemotherapy and additionally in the end of concurrent chemoradiotherapy. The CEC values of the observation group showed significant statistical differences (*p* < 0.05) before or after different therapies, whereas those data in the control group were not statistically different. And, the mostly importantly, the CEC values in the observation group and control group turned out a statistical difference. The combination of endostatin and chemoradiotherapy significantly reduced parameters of peripheral blood CECs in these patients. According to the CEC parameters' variety that we observed in the combined therapies, this study demonstrated that the CECs might be a clinical clue to evaluate this antiangiogenic chemoradiotherapy. And the clinical value of CECs will be further determined along with increasing comparative studies and clinical long-term efficacy observation.

## 1. Introduction

Nasopharyngeal carcinoma (NPC) is a sort of epithelial malignancy that occurs frequently in Southeast Asia and North Africa (1). Studies indicate that genetic, ethnic, and environmental factors may jointly influence the pathogenesis of NPC (1–3). The current treatment for nasopharyngeal carcinoma is mainly radiotherapy. However, a large proportion of patients will experience local recurrence or distant metastasis after treatment (3). The Chinese Society of Clinical Oncology (CSCO) clinical guidelines for the diagnosis and treatment of nasopharyngeal carcinoma (2021) adds grade I recommendations in first-line treatment for recurrent/metastatic nasopharyngeal cancer: cisplatin +5-fluorouracil (5-FU) + local radiotherapy and new recommendation for grade III: cisplatin + gemcitabine + endostatin (recombinant human endostatin) (4). Folkman proposed the theory that tumor growth and metastasis are reliant on angiogenesis in 1971 (5). This theory suggested that curbing tumor angiogenesis is the key factor to inhibit tumor growth and metastasis (5). Recombinant human endostatin has the functions of inducing apoptosis of vascular endothelial cells, inhibiting tumor angiogenesis and inhibiting cell proliferation and migration (4).

Peripheral blood is a convenient biopsy sample that can be obtained without trauma. Peripheral blood is used for biomarker detection. CECs are a kind of vascular endothelial cells free in peripheral blood. These cells are associated with angiogenesis and the growth and metastasis of tumor, deemed as the target of angiogenesis inhibitors and the biomarker to appraise therapeutic efficiency. Moreover, numeric alteration of CECs is also a biomarker to estimate the damage of vascular endothelium. An essential process in tumorigenesis and metastasis is angiogenesis (6, 7). The numeric alteration of CECs is a favorable predictive factor to appraise angiogenesis and prognosis (8). Recombinant human vascular endostatin is currently a widely applied injection in clinical, but its treatment outcome is hard to trace. Numeric increasement of the CECs in human lymphoma xenograft mouse models was positively correlative with tumor load, and it also implied its relationship with tumorous occurrence and development (9). On the basis of the both comparison and observation into the CEC alteration in patients' peripheral blood samples during our combined treatment, we elucidated the clinical significance of peripheral blood CEC detection in antiangiogenic chemoradiotherapy.

## 2. Patients and Methods

### 2.1. The Patients and Their General Information

Our subjects were the patients who were treated in the Head and Neck Oncology Department of Guizhou Province Cancer Hospital, dating from May 9, 2012 to March 10, 2013. Here is the clinical trial registration: Chi CRT-ONRC-12002394.

The trial was approved by the ethics committee at Guizhou Province Cancer Hospital. Inclusion criteria were as follows: male or female, the ones aged from 18 to 70 who were volunteered and offered a written consents for medical treatment; the one whose carcinoma was diagnosed as differentiated or undifferentiated type of nonkeratinizing nasopharyngeal carcinoma; their clinical stages were about at III-IVa and IVb (basing on 2010 UICC); KPS > 70, life expectancy ≥ 6 months; and whose white blood cell, hemoglobin, platelet, and liver and kidney function values were within the normal reference value range. No serious complication was demanded, such as hypertension, diabetes, coronary heart disease, and mental illness; this treatment was the first course of treatment (no history of head and neck radiotherapy, no history of concurrent radiotherapy and chemotherapy, no history of chemotherapy within 3 months). Exclusion criteria were as follows: the ones were with serious and uncontrolled medical illness or suffering major organ failure. All patients in this study were not randomly divided, and another 47 cases of the patients were enrolled as Clinical study control.

### 2.2. Inductive Chemotherapy

Both the control group and observation group were commenced with a two-cycle (with a cycle of 21 days) inductive chemotherapy TP (docetaxel, Jiangsu Aosaikang Pharmaceutical, E1203012) + cisplatin (Shandong Qilu Pharmaceutical, 2A1A1202011A): a one-day intravenous drip of 75 mg/m^2^ docetaxel, and the subsequent intravenous drip of 80 mg/m^2^ cisplatin over the next three days was conducted.

Eight days after inductive chemotherapy, the observation group was additionally treated with an intravenous drip of 7.5 mg/m^2^/day recombinant human endostatin (Endostar Jiangsu Mr. Pharmaceutical, 201201001), and this treatment lasted for 14 days (a cycle of the treatment).

### 2.3. Concurrent Chemoradiotherapy

Both the control group and observation group were given a cisplatin (intravenous drip of 80 mg/m^2^ cisplatin was given on the first day and second day of the therapy) concurrent chemotherapy after first-day radiotherapy. The observation group was treated with an additional recombinant human endostatin intravenous drip with the dose of Endostar 7.5 mg/m^2^/day two weeks after the concurrent chemoradiotherapy, and this treatment lasted for a cycle of 14 days.

### 2.4. Radiotherapy

Both the control group and observation group were given intensity modulated radiation therapy (IMRT) (TOSHIBA Atlas, Japan) targets, and therapeutic dose was shown in report (10).

### 2.5. Flow Cytometry Detection of CECs

The isotype control of each sample was performed to eliminate the interruptions from background and cell immunofluorescence. Two clean sterile test tubes were tagged as control tube and experimental tube. The tube tagged as control was added with 100 mL whole blood and 20 *μ*L isotype antibody, prepared as the control. The tube tagged as experimental was added with 100 *μ*L whole blood and 20 *μ*L CECs detection antibody. Both the tubes were kept at room temperature in the dark for 15 min, which were subsequently added with 800 *μ*L 1× hemolysin and subjected to a room-temperature 5 min incubation in the dark. Then, these tubes were incubated in a water bath at 37°C for 5 min and centrifuged at 1000/min. The leftovers in these tubes were rinsed with PBS twice and resuspended. The on-machine processing was carried out on a flow cytometer (BD, USA). 1 × 10^4^ mononuclear cells were collected in each sample, whose data were analyzed with BD FACSDIVA analysis software. FITC-anti-human CD3*ε* monoclonal antibody, PE-anti-human CD146 monoclonal antibody, FITC-anti-human IgG1 antibody, and PE-anti-human IgG2a antibody were purchased from BD PharMingen, USA. Three independent replicates were performed.

These white blood cells varied in size and complexity within the nucleus, which were categorized into three populations basing on FSC/SSC collection chart, from left to right: lymphocyte population, monocyte population, and granulocyte population. A circle gate analysis was performed on lymphocytes and monocyte populations (i.e., mononuclear cell populations). FITC-anti-human IgG1 and PE-anti-human IgG2a were deemed as isotype controls and adjusted the voltage and compensate: the number of CECs = CD3 − CD146 + per 10,000 mononuclear cells.

### 2.6. Observation Indicators and the Follow-Up

Peripheral blood CEC values of patients in the observation group and treatment group were obtained and recorded as above. In the observation group, one case (4%) of patients with cardiac adverse reactions occurred. The remaining adverse reactions were mainly nausea and vomiting (16%) associated with chemotherapy. The content of the follow-up included the curative efficacy at 3 months, 1 - and 3-year progression-free survival, and overall survival. We also followed up patients by phone every 3 to 6 months and notified them to return to the hospital for review.

### 2.7. Statistical Methods

SPSS 22.0 was applied for the data statistical analysis in this experiment. Measurement data were expressed in form of mean ± standard deviation or median (upper and lower quartile), and count data were expressed in the number of cases (percentage). Chi-square test was applied for the comparison onto T stage, N stage, gender, age, pathological type, and effective rate between groups. The changes of CECs in the control group and the observation group before and after treatment were compared by paired *t*-test. The cumulative overall survival (OS), disease free survival (DFS), progression-free survival (PFS), and distant metastasis-free survival (DMFS) at 1, 3, and 5 years were calculated by the Kaplan-Meier method to evaluate progression-free survival and overall survival. Log-rank test was used for comparison between groups to draw survival curves.

## 3. Result

### 3.1. Clinical Characteristics of the Patient

There were 25 patients, aged from 31 to 70, in our treatment group, made up of 7 female and 18 males with a median age of 52 years old. Pathological types were made up of 5 cases of the nonkeratinized differentiation and 20 cases of the nonkeratinized undifferentiation. The control group was made up of 6 female and 16 males, with 22 cases of patients aged from 30 to 70 in total with a median age of 47 years old. Pathological types were made up of 3 cases of the nonkeratinized differentiation and 19 cases of the nonkeratinized undifferentiation. There were no significant differences in age, gender, pathological type, and clinical stage between the two groups (Table 1).

### 3.2. The Numeric Alteration of CECs in the Observation Group

There was a declining trend of the CECs in the observation group. The alteration of the treatment group was shown in Figure 1. The value of CECs before induction was 14.96 ± 7.62, and after induction was 10.16 ± 5.14, resulting in their difference statistically significant (*t* = 2.61, *p* = 0.037). The value of CECs before induction was 14.96 ± 7.62, and after radiotherapy was 5.84 ± 6.76, having their difference statistically significant. The value of CECs after induction was 10.16 ± 5.14, and that after radiotherapy was 5.84 ± 6.76, making a statistical significance (*t* = 2.54, *p* = 0.004).

### 3.3. The Numeric Alteration of CECs in the Control Group

There were no significant alterations in CEC values revealed in the observation group (Figure 1). In the control group, the value of CECs before induction was 13.77 ± 6.60, and after induction was 12.59 ± 6.24, showing no statistical significance (*t* = 0.09, *p* = 0.515). The value of CECs before induction was 13.77 ± 6.60, and the value after radiotherapy was 10.27 ± 5.02, representing no statistical significance (*T* = 0.31, *p* = 0.057). The value of CECs after induction was 12.59 ± 6.24, and after radiotherapy was 10.27 ± 5.02, turning out a statistical insignificance (*t* = 0.21, *p* = 0.204). CEC value of the observation group and in the control group after radiotherapy was 5.84 ± 6.76 and 10.27 ± 5.02, showing a statistical significance (*t* = 2.57, *p* = 0.001). It demonstrated that endostatin combined with inductive chemotherapy and concurrent radiotherapy significantly reduces the number of CECs in the blood of patients.

### 3.4. Follow-Up Results

The effective rate of treatment in the whole group reached 100%, and the CR rates (3 months after concurrent radiotherapy and chemotherapy) of the observation group and the control group were 60% and 50%, respectively (*t* = −1.725, *p* = 0.091). There was no statistical distinction within groups; the CR rates of the observation group and the control group after 1 year were 100% and 95.45%, respectively (*t* = 1.000, *p* = 0.332), having no statistical significance. The last follow-up was on July 30, 2018, with a median follow-up of 70 months, and the follow-up was 100% completed. Our results turned out that there were 11 deaths from various causes: 5 deaths in the observation group and 6 deaths in the control group; 1-, 3-, and 5-year OS, DFS, PFS, and DMFS in the observation group had survival advantages over those in the control group, but there was no statistical significance in the two groups (Table 2). The survival curve was shown in Figure 2.

## 4. Discussion

The mainstream treatment for advanced local nasopharyngeal carcinoma patients is a comprehensive treatment combining with radiotherapy, chemotherapy, and targeted therapy, which greatly improves patients' five-year survival rate and especially has that of the advanced local nasopharyngeal carcinoma (stages III and IVa) which reach nearly 80%. Failure of nasopharyngeal carcinoma IMRT mainly attributes to the distant metastasis of this cancer (11–14). Therefore, controlling local recurrence and distant metastasis might ensure the long-term survival of patients.

Short-term effective rate of recombinant human endostatin combined with induction chemotherapy and sequential concurrent chemoradiotherapy in the treatment of advanced local nasopharyngeal carcinoma was higher than that of induction chemotherapy and sequential concurrent chemoradiotherapy (10). Antiangiogenesis therapy normalizes tumor angiogenesis and alleviates tumor hypoxia, thereby elevating tumor radiotherapy and chemotherapy sensitivity (15, 16).

Antitumor neovascularization is an important aspect of targeted therapy, but the evaluation standard for tumor efficacy is mainly the evaluation to chemotherapy drugs' efficacy (17–19). Antiangiogenic drugs act on the blood vessels of tumors, and most of them cannot quickly shrink tumors, because tumorous volume change often comes later than blood supply inhibition. Therefore, the mere evaluation to tumor volume is not objective enough, which makes the current evaluation to antiangiogenic drugs still limited. The evaluation to antiangiogenesis effect mainly includes imaging examination, biomarker detection, morphological examination, and clinical symptoms.

In addition to vascular endothelial growth factor, the related biomarkers also include peripheral blood circulating endothelial cells. It has been found that the binding of vascular endothelial cell-specific heparin to growth factors can promote the formation of new blood vessels in vivo (20, 21). The high expression of VEGF is regarded as one of the potential markers of early metastasis of nasopharyngeal carcinoma, which often indicates lymph node metastasis, recurrence, and poor prognosis of nasopharyngeal carcinoma. The CECs in lung cancer patients reflected lung cancer angiogenesis and were used to judge the prognosis (11). The number of CECs in the blood of patients with head and neck tumors was also increased, which is associated with VEGF (22). Goon et al. compared the number of CECs detected through magnetic separation and flow cytometry, and they found that in the case of specific CEC phenotype, flow cytometry was more accurate in detecting the number of CECs (23).

This study was implement via the added recombinant human endostatin to the usual treatment of patients with advanced local nasopharyngeal cancer, and our results turned out that the CEC value in the observation group before the inductive chemotherapy was 14.96 ± 7.62, and after concurrent chemoradiotherapy was 5.84 ± 6.76, showing a notable numeric alteration that the difference is statistically significant; however, the value of CECs in the control group was 13.77 ± 6.60 before induction chemotherapy and 10.27 ± 5.02 after concurrent radiotherapy and chemotherapy, and there was no obvious difference between the pre and the post, where the difference was statistically insignificant (*p* = 0.057). By comparing the values of CECs at the end of treatment, we found that the CEC value in the observation group was notably lower than the control group with the difference statistically significant (5.84 ± 6.76, 10.27 ± 5.02, *t* = 2.57, *p* = 0.001). Our results are consistent with those reported by Lee et al. (3), and it shows that endostatin combined with inductive chemotherapy and concurrent radiotherapy significantly reduces the number of CECs in the patient's blood, indirectly illustrating potential efficacy of recombinant human endostatin in the treatment of nasopharyngeal carcinoma. Previous research reported that CECs are increased in the blood of cancer patients and correlate with angiogenesis, therefore potentially serving as a biomarker to determine progressive disease, prognosis, and response to therapy (24, 25). In the long-term follow-up, we found that the observation group showed a slight survival advantage trend of OS and PFS, but there was no statistical difference. Guan et al. confirmed that the CR rate of recombinant Endostar and radiotherapy for advanced, locally recurrent nasopharyngeal carcinoma could reach 90.9% (26).

The combination of endostatin and chemoradiotherapy reduced parameters of peripheral blood CECs in these patients. This study demonstrated that the CECs might be a clinical clue to evaluate this antiangiogenic chemoradiotherapy. The limitation of this study was the number of cases that is relatively small. There were 11 deaths from various causes: 5 deaths in the observation group and 6 deaths in the control group in our study. This may be why CR reached 100% after 1 year. Considering that the number of patients in the group may be less, no statistical difference was shown. The shortcomings of this study lie in the nonrandomized comparative study to single-center small samples, and the number of cases is relatively small. Further clinical application of this study needs to be confirmed in a large multicenter phase III clinical study.

## 5. Conclusion

In this study, we found that concurrent chemoradiotherapy combined with endostatin effectively decreases the CEC number in peripheral blood of patients with advanced local nasopharyngeal carcinoma versus the control group. Through long-term follow-up of patients, we can see the trend of survival benefits. We believe that the detection to CEC numeric alteration in peripheral blood is potentially significant clinical measures to evaluate the efficacy of antiangiogenesis combined radiotherapy and chemotherapy.

## Figures and Tables

**Figure 1:** The changes of CECs during the treatment. ^∗^*p* < 0.05, ^∗∗^*p* < 0.01.

**Figure 2:** The survival curve of OS, DFS, PFS, and DMFS.

**Table 1:** The clinical characteristics of 47 nasopharyngeal patients.

Characteristic	Treatment group	Control group	*p* value
Gender			0.956
Male	18	16	
Female	7	6	
Age^∗^			0.196
Range	31-70	30-70	
Median	52	47	
Pathological type^∗∗^			0.849
Undifferentiated type	20	19	
Differentiated type	5	3	
Clinical stages△			1.000
*ΙΙΙ* stage	2	2	
*Ι*V stage	23	20	

Note: ^∗^ in age, △ 2010UICC stage, ^∗∗^ nonkeratinizing cancer.

**Table 2:** The survival comparison between the two groups.

Items	Treatment group	Control group	*χ* ^2^/*Z* value	*p* value
*N*	25	22		
OS			0.291	0.589
1 year	92%	90.9%		
3 years	88%	77.3%		
5 years	76%	72.7%		
DFS			0.203	0.653
1 year	92%	90.9%		
3 years	76%	77.3%		
5 years	68%	67.7%		
PFS			0.046	0.830
1 year	92%	90.9%		
3 years	80%	81.8%		
5 years	68%	72.7%		
DMFS				
1 year	92%	90.9%	0.136	0.712
3 years	84%	77.3%		
5 years	76%	68.2%		

## Data Availability

The data used to support the findings of this study are included within the article.
